# Accessibility of Urban Nonprofit Public Nursery Services Based on Big Data

**DOI:** 10.1155/2022/9775524

**Published:** 2022-07-16

**Authors:** Yi Li, Xiaoli Deng, Shan Liao, Xiaoli Liang, Hongyan Wang, Hua Fang, Zhen Ai, Pei Chen, Xiangeng Zhang

**Affiliations:** ^1^Department of Scientific Research, Sichuan Vocational College of Nursing, Chengdu 610100, China; ^2^Department of Nursing, Sichuan Vocational College of Nursing, Chengdu 610100, China; ^3^Sichuan Ambay Medical Technology Co Ltd, Chengdu 610000, China; ^4^Academic Administration, Sichuan Vocational College of Nursing, Chengdu 610100, China; ^5^Research Center for Higher Education Development, Sichuan Vocational College of Nursing, Chengdu 610100, China; ^6^Tangwai Experimental Kindergarten, Chengdu 610000, China; ^7^Chengdu, Institute of Biological Products Co Ltd., Chengdu 610000, China; ^8^Sichuan Nursing Vocational College 173 Longdu South Road Longquanyi District, Chengdu 610000, China

## Abstract

In today's society, the pressure of family care is increasing and people's demand for childcare services is increasing. At the same time, the government also pays more attention to the problem of 0 ∼ 3-year-old infant care services which are desperately needed in every society throughout the world. General studies have been carried out in literature where results show that in families with only one child, long working hours and with more than two children, the three factors of children's age gap, attention to nursery facilities, attention to environment and food safety have a negative impact on people's demand for nursery services. From these studies, we have extracted three vital factors that have a positive impact on people's demand for childcare services: grandparents' help to take care of children, parents' age, and psychological tolerance of childcare service fees. In this paper, we have utilized one of the most commonly used methodology, i.e., big data, to smoothly resolve the accessibility issue of urban non-profit public nursery services. In order to verify and evaluate our claim, we have implemented the proposed scheme and compared the results which shows that exceptional performance of the propose scheme.

## 1. Introduction

In recent years, the national policy on family planning has been continuously relaxed. It is an interesting domain which got importance due to mass increase in the population of the world and family planning is one of the most important methodologies for controlling it. It is defined as “the exercise to develop a proper management or control policy to ensure how the number of children has to reduce, preferably one, and the intervals between their births (minimum possible duration or permanent), especially through the contraception or voluntary sterilization.” Although the current laws in some areas stipulate that social maintenance fees shall still be levied for those who have more than two children, there have been significant changes compared with the previous policies of “double only two children” and “single two children”. After the implementation of the “comprehensive two child” policy ①, the increase of China's population fertility did not meet expectations [1]. Other studies ④ show that there is a close relationship between fertility and the allocation pattern of educational resources, and infant education plays a very important role in educational resources. The lack of educational resources and differential allocation will inevitably bring competition for educational resources and also bring great pressure to children's parents. Under this condition, people put more energy and financial resources into limited educational resources by reducing fertility, in order to get better educational resources and less pressure.

“No one takes children” has also become one of the important factors affecting the fertility rate due to the lagging development of educational resources. According to the survey ⑤ of fertility willingness released by the National Health and Family Planning Commission in 2015, 74.5%, 61.1%, and 60.5% of the factors are unwilling to have a second child because of economic burden, too much energy, and no one to look after them, respectively. A survey conducted by the NLD shows that 68.1% of mothers who have given birth to one child but do not intend to have a second child are because their children are unattended ⑥. In 2016, the China Women's Federation and Beijing Normal University issued a survey report on the impact of the implementation of comprehensive two child education on family education. The report showed that 53.3% of one child families had no intention of having two children. The survey found that the four public service resources of education, medical treatment, health, and living environment were the most important factors affecting the decision-making of two children. With the development of society, infant care has gradually become a more significant social problem. Infant care is not only the responsibility of the family, but also needs the support of the government and the supply of public services [2]. Therefore, in recent years, infant public care services have attracted more and more attention.

The employment rate of women in cities is higher than before, and under the influence of the new social culture, they pursue a higher quality of life. At the same time, they also bear greater life pressure, and the energy and time of childcare are obviously affected ①. At the same time, these women are also more expected to return to the workplace. For ordinary families, the average marriage age has gradually increased in recent decades, resulting in grandparents' increasing age when looking after infants and young children, a relative decline in their ability to take care of children, and a relative increase in the pressure on grandparents to take care of young children [3]. These reasons may lead to a decrease in grandparents' willingness to take care of young children ②. Children's early education and care is the basis for learning cognition and various skills. Children's later development largely depends on the quality of children's care and education ③. Therefore, parents have higher and higher requirements for the quality of their children's care. They hope that their children can learn more scientific knowledge and skills and develop their abilities appropriately while being taken care of. This is obviously not available in traditional care, and public childcare services have these advantages and can meet the needs of parents [4].

In October 2017, in the report to the 19th National Congress of the Communist Party of China, it was mentioned to implement “education for children, learning and education,” and put “education for children” in the first place in the progress of people's livelihood. However, at present, China's infant care services are still seriously insufficient [5]. According to the data released by the National Health and Family Planning Commission, the enrollment rate of 0–3-year-old infants in various kindergartens in China is only 4%, and the enrollment rate of urban infants under the age of 3 is less than 10%. Recent surveys in Changsha, Yongzhou and other places also found that 90% of parents believe it is necessary to let children participate in childcare and early education, but nearly half of them did not participate because of economic and social reasons ⑤. Therefore, facing the huge gap, the establishment of a complete public childcare service system is imminent.

As for the demand for childcare services, a large number of scholars have studied the macro environment: first, women's market participation has increased. Since the marketization, women have gradually been liberated from the family and participated in the labor market. As a result, women are facing the conflict between childcare and job choice, which also increases the pressure on them to take care of children and forces them to find other ways of infant care. Second, population aging and care deficit. Facing the problem of population aging, the state has issued policies to delay the retirement age [6]. At the same time, with the improvement of grandparents' requirements for the quality of life of the elderly, they prefer to enjoy the life after retirement rather than help take care of their grandchildren, which makes there less infant care resources from grandparents. Third, population mobility and miniaturization of family structure. With the reform and development of the economic system, the scale of population flow is unprecedented, and the family tends to be smaller. The parents need to go out to work, and the grandparents and core families live in different places, which increases the childcare cost within the family, leads to the lack of “helpers” and the obvious weakening of the family's care function [7].

With the strong support of government policies and the strong demand of the people, the establishment of the childcare service system should receive more attention and research, however, this research filed is still in its infancy and careful attention is required from the academia and research organization. Therefore, it is necessary to explore the influencing factors of the people's demand for childcare services.

To address the issue mentioned above, we have developed and reported a big-data-enabled system for the accessibility of urban non-profit public nursery services especially those which are required to be ensured by the concerned government. Additionally, we have devised a methodology that a government will ensure that these services and measures are needed to be taken on timely basis.

The rest of the paper is organized as given below.

In the subsequent section, an extensive review of the available techniques, preferably those which are closely linked to the problem at hand, is presented along with various problems in the existing approaches are highlighted. In the next section, the proposed methodology is well explained in various sections and subsections along with how these issues could possibly be resolved. Results and discussion are provided in a separate section. Finally, concluding remarks are provided in the last section of the paper.

## 2. Related Work

In recent years, with the relaxation of the national fertility policy, more and more families have entered the ranks of “two child families”. With the emergence of various parenting problems, the Chinese government is also actively introducing various parenting policies. Experts and scholars in many fields such as education, sociology, and economy are also actively exploring, and the “public childcare service” has gradually become a hot spot in the academic community.

Different scholars have different views on the definition of childcare service. ③ Childcare is an alternative service. When families cannot take care of infants and young children for some reason, childcare services can take care of infants and young children instead of families. At the same time, childcare services can significantly reduce the rearing pressure of some families, liberate family productivity, and promote social development. [4] It is considered that nurseries are services to assist families in providing care, health care, and infant development experience. [5] Childcare is a variety of day care and arrangements chosen by the parents for their children. The purpose is to enable infants and young children to be cared for, protected, and fully educated. [6] The right to care is an important part of civil rights. The essence of childcare is the guarantee of the right to care.

As for the function of childcare services, Peng Shuhua believes that childcare services can not only promote women's employment, but also enhance family stability. ② infants aged 0–3 are in the early stage of life cycle. Their life experience and experience during this period have an important impact on personality and intelligence. Good public care services are conducive to the development of infants and young children and the formation of good habits. ③ the “elderly floating” group has difficulties and pressure in infant care. A perfect social infant care service system is conducive to liberate the elderly who care for their grandchildren and reduce the burden of the elderly group. ④ the survey found that in the case of a shortage of public childcare services, urban women who have two children and take care of children aged 0–3 have a higher proportion of family impact on work, a larger gender gap, and some women are forced to interrupt their work. The perfect public childcare service system is conducive to liberating women's productivity, narrowing the gender gap, and reducing the impact of work on families.

For the discussion of the mode of nursing service, ⑤ the ways and methods of providing services are different for the nursing institutions established by different subjects. According to the different supply subjects and scale, nurseries are mainly divided into family nurseries, enterprise nurseries, community nurseries, institutional nurseries, and PPP nurseries. ⑥ taking the new public service theory as the framework, this paper puts forward seven elements: concept, mode, project, specification, mechanism, effect, and policy to identify and classify the practice mode of infant care service in China.

Infant care services originated in western countries. In the 1950s and 1960s, the birth rate in western countries increased significantly after the war, which led to the increasing inability of traditional families to take care of infants. At this time, a large number of socialized childcare institutions appeared, and childcare services came into being. At present, the research literature on international childcare services mainly includes the introduction of childcare service model, development experience, and evaluation of treatment in childcare institutions in foreign developed countries, but there are few related in-depth discussions [8].

Some social democratic countries in northern Europe pursue the value orientation of inclusive development, as well as the principle of highly non-commodity delimitation and universalism. In these countries, the government provides infant care services, advocates the socialization of the family cost of raising, creates a social environment suitable for taking care of children, and the government provides various needs in the process of infant growth. This welfare policy can not only ensure the family's ability to raise infants and young children, but also reduce the burden of family care for infants and young children through free choice ①.

In countries like Norway and Sweden, each and every woman is allowed and encouraged, i.e., through various means, either to take part in the working environment where men are supposed to work. As we know that various hurdles have been reported but participation of the women in the working environment especially under the concerned policy is very encouraging. Additionally, these type of services removes the barriers for women which are in different societies throughout the world. Apart from this, these countries have specifically contributed to the education sector where it is ensured that education provided by these countries is generally integrated education, that is, the combination of trusteeship and early education.

Some other countries in Europe pursue the value orientation of filling vacancies, survival, and re-family. These countries attach great importance to the maintenance of traditional family relations and regard taking care of children as the responsibility of mothers. The government will take care of children only when the family is unable to take care of infants and young children. The service models of these countries emphasize the family's ability to support. In this case, the development of public childcare services is greatly limited. It is difficult for general infants to obtain childcare opportunities, and women's rights and interests have also been hurt to some extent. This category includes Germany, Italy, and other countries. In such countries, the way of childcare is generally phased service. For example, in Germany, infants aged 0–2 only receive childcare services, and infants aged over 3 receive early education at the same time.

In addition, some developed countries pursue the value orientation of filling vacancies and survival, but from the perspective of family, they pursue the concept of de-familialization. The type of social welfare in these countries is generally liberal welfare. These countries emphasize the regulatory role of market mechanism. The state only provides necessary help to poor families and only guarantees the minimum level of welfare. Few infants and young children finally receive the childcare services provided by the state ③. Like the Nordic countries, these countries generally advocate the principle of educational integration, and children can receive early education while receiving custody services [9].

Foreign childcare services developed earlier, and both the development of policy system and the large-scale development of childcare institutions are relatively perfect. Compared with domestic, foreign public childcare services started earlier. The American Association of Preschool Education issued a certification standard for high-quality childcare institutions in 1984. Its core idea—the development of suitability education has had a wide impact all over the world. In view of the differences in the development of childcare services at home and abroad, Qiu Baili ④ through the comparison between the kindergarten evaluation standards formulated in Zhejiang, Jiangsu, and Shanghai and the certification standards of high-quality childcare institutions formulated by the American Preschool Education Association believes that there is still a certain gap between China and foreign advanced educational ideas [10]. Reference [11] believes that foreign values are more advanced, the system is more perfect than that is in China, there are laws with high feasibility to provide protection, and a variety of allowances to provide meticulous care for infants and young children and economic support for parents. Humanized welfare policies and all-round childcare services can meet the different needs of all kinds of children and families to the greatest extent. Reference [12] through the comparison with EYFS nursery institutions in the UK in terms of examination and registration, teacher-child ratio, qualification, and training, it is considered that there is still room for improvement in the supervision and implementation, teacher-child ratio, employee education, and training mechanism in China's preschool education.

Generally speaking, the foreign public childcare service system is not perfect, and there are also problems such as the distribution of rights and responsibilities, financial investment, the qualification of institutions, and educational security personnel [13]. However, many of its systems and concepts are more advanced and worthy of our study.

## 3. Childcare Services

Childcare service is a part of children's welfare. It is transformed from the word “childcare.” At first, it means “entrusted parenting,” that is, to entrust infants and young children to people or institutions other than family caregivers for parenting and care. With the changes of the times, people's demand for childcare services is not only satisfied with the initial upbringing and care, but also organically combines “education” and “maintenance,” The United Nations defines childcare services as the care and education received by children outside the family from groups or institutions. In OECD countries [14], however, it is important to note that childcare is not only concerned with the outside environment as various authors have perceived it differently such as childcare services start from the home, this is actually the thought of certain group of authors. Additionally, a certain class of authors believe that childcare service starts exactly when a child has to interact outside his/her home. It is considered that all services including formal and informal care and education for preschool children are childcare services. Public childcare service is a kind of childcare service, which refers to the childcare service provided or participated by the government or public forces. In China, the service content mainly includes early education and nursing. For the definition of infant age, infants aged 0–3 are generally regarded as the research object of public childcare services in China. In fact, in more developed big cities, the strict sense of nursery institutions are mainly kindergartens, community childcare centers built by the government, and internal custody centers established by some enterprises. Some enterprises participate in the provision of nursery services in the form of internal employee welfare. However, the market-oriented force that really takes the supply of childcare services as the core operation and management business is still in the blank stage, and the real market-oriented supply of childcare services is relatively lacking ①.

It is to be noted that generally the public childcare service is how education is provided to these children. However, in this paper, childcare service has been referred to as environment where education along with other necessary services are provided especially by the concerned government. Additionally, it is to be noted that it is the responsibility of the concerned government departments to ensure supply of subjects directly or to the childcare institutions directly or indirectly. However, this entire process is desperately needed to be managed by the government for 0–3-year-old infants, including daily life care, nutrition matching, habit formation, and early education, in order to achieve their development, learning, and growth goals. Finally, if some of these services are missed or not provided on a timely basis then it may affect the life of the infants.

## 4. Data Description and Model Setting

Generally, we know that for providing a big-data-enabled model, data is needed. As we have described below, a dedicated survey was conducted to collect the desired data needed for the verification of the proposed study and to be in a better position to enable or at least develop a system where childcare services are ensured by the concerned government.

### 4.1. Data Sources

The data used in this article comes from the data obtained from the extensive survey conducted by the research group of Jiangsu Institute of social security from January 2019 to March 2019. The research group took married young people aged 20 ∼ 40 as the survey object, and collected the basic information of the respondents and their families, the survey of the respondents' fertility willingness and fertility, and the survey of infant rearing and childcare services to study the residents' infant rearing and childcare services. A total of 683 valid questionnaires were collected, involving 93 cities in 17 provinces such as Jiangsu, Anhui, and Guizhou. As the research objects are concentrated in the respondents and their families with infants aged 0 ∼ 3 years, the survey data corresponding to the families with the youngest child aged 3 years and below were selected. At the same time, after deleting the missing data and abnormal data, a total of 190 valid sample data were obtained [15].

### 4.2. Variable Description

In this study, proper description of the various variables which are being utilized such as explanatory variables. These variables were used to explain whether there is a demand for childcare services in a particular region; likewise, the explanatory variables are used to represent various possible factors that affect people's demand for childcare services. Various effects of these factors are family income, the current care mode of children, the age difference of children in multi-child families, whether there is an only child in the parents' generation, whether they live with their grandparents now, the working hours of parents, the distance between childcare institutions and home. The characteristic variables of nursing institutions, such as the charging level of nursing institutions and the charging level of institutions they can bear.

### 4.3. Model Design

In order to calculate the regression model, it is assumed that:

(1) $$\begin{array}{c} f\_ty=\alpha +\sum_{i=1}^{n}\beta_{i}x_{i}+e_{i}. \end{array}$$

Where, *if*_*ty* is the basis of decision-making, *if*_*ty*  = 1, representing the need for childcare services; *if*_*ty*  = 0, which means no nursery service is required. *x*_*i*_ is the variable for each sample, *β*_i_ is the parameter corresponding to each variable, *α* is the intercept term, *e*_*i*_ is the random error term obeying the standard normal distribution. *x*_*i*_ impact on the demand for childcare services is determined by formula (2):

(2) $$\begin{array}{c} P\left(if\_ty=1|x_{i}\right)=P\;\left(if\_ty=\alpha +\beta_{i}x_{i}+e_{i}>0\right)\\ =P\left(e_{i}\leq \alpha +\beta_{i}x_{i}\right)=F\left(e_{i}=\alpha +\beta_{i}x_{i}\right). \end{array}$$

Logistic distribution:

(3) $$\begin{array}{c} P\left(if\_ty=1|x_{i}\right)=\frac{1}{1+\left(\exp^{-\left(\alpha +\beta_{i}x_{i}\right)}\right)} \end{array}$$

When *α*+*β*_*i*_*x*_*i*_ tends to infinity, *P*(*if*_*ty*=1*|x*_*i*_) is infinitely close to 1, whereas, when *α*+*β*_*i*_*x*_*i*_ is infinitely small, *P*(*if*_*ty*=1*|x*_*i*_) is close to 0.

## 5. Analysis of Empirical Results

Analysis is one of the methods which is available in literature and are used to ensure applicability and feasibility of a newly developed system in the expected environment where the proposed system is supposed to be deployed.

### 5.1. Empirical Analysis

Logistic regression was used to analyze the impact of different factors on whether people choose childcare services. As shown in Table 1, the impact of parents being the only child on the choice of childcare services shows that the impact of respondents being the only child on the choice of childcare services is negative, and the probability ratio of respondents choosing childcare services for the only child is 0.486 times that of the respondents not being the only child, The probability ratio of respondents choosing childcare services for their only child is 0.456 times that of respondents whose spouse is not the only child, and the probability ratio of families with both husband and wife being the only child is 0.358 times that of families with both husband and wife not being the only child. It fully shows that families with only one child are less likely to choose childcare services. At the same time, when controlling the variable that the respondents are the only child, the regression results show that the longer the respondents work at home, the less inclined they are to choose childcare services. The probability ratio of choosing childcare services relative to not choosing childcare services decreases by 2% for each additional hour of family working time. Generally, in our society, we have observed that for those couples, whose working schedule is hard and comparatively longer than usual, it is high likely that they will surely require services, i.e., help in most of the case, to ensure proper caring of their infants. This could possibly be ensured through either a servant or if there are other family members like parents of the husband or wife or both, however, this is very rare in different societies and thus other alternatives are needed to be provided. In the situation that the concept of childcare has not been formed and the development of the childcare market is not perfect, the first choice is the help of grandparents, so that people will not choose to buy childcare services first. However, this does not mean that with grandparents to help take care of children, there is no need for childcare services. The probability of families with parents and grandparents taking care of their children choosing childcare services is 1.279 times higher than that with only parents.

Table 2 shows that when controlling the variables such as the age of respondents, the age of the first child in the family, whether the parents are the only child, and whether the grandparents live together, it is found that the greater the age difference between the second youngest child and the youngest child, the less likely they will choose childcare services. The data show that the age difference between the second youngest child and the youngest child has an impact on whether the family chooses childcare services at a significant level of 5%. When the age difference increases by one year, the probability of families choosing childcare services decreases by 251% compared with not choosing childcare. For families with more than two children, the greater the age difference between the second child and the youngest child, the less pressure the family has to take care of. When the age of the respondents increases by one year, the probability of requiring childcare services increases by 95% compared with not requiring childcare services.

Table 3 shows the impact of the situation of childcare institutions on people's demand for childcare services. The data in the table shows that people who care about the distance between the nursery institution and their home need more nursery services. People who care about the facilities, environment, and food safety of care institutions do not need care services compared with those who do not care much. People who care about the fees charged by nursery institutions have more demand for nursery services. People who have a higher bearing on the charge level of childcare services are more likely to choose childcare services.

### 5.2. Result Analysis

The discussion from the micro-personal aspect mainly focuses on the following aspects: on the one hand, the requirements for the improvement of education quality are in conflict with the educational ideas of grandparents. After the introduction of the two-child policy, the grandparents are old, and their enthusiasm for the care of their grandchildren is not high, and people's professional requirements for the level of infant care are gradually improving. Even if grandparents are willing to take care of their children, in the face of the conflict of parenting concepts of grandparents when taking care of their grandchildren, more and more parents refuse the care of their grandparents. On the other hand, the parents work intensively and lack professional parenting knowledge. Parents face problems such as high work intensity and insufficient parenting experience and are unable to give scientific, full, and all-time care to infants and young children. Through the above analysis, it is not difficult to draw a conclusion: people's demand for childcare services exists in reality, and the demand is large. According to the data released by the National Health Commission, the current shortage of childcare services in China is very serious. The enrollment rate of 0–3-year-old infants in various childcare institutions in China is only 4%, far lower than the proportion of 50% in some developed countries ①. According to Wang Hui's research results, the enrollment rate of children under the age of 3 in the Chinese cities is less than 10%, and there are differences among provinces. There is a great difference between the expectation of local people and the actual proportion of local children. Among them, 90% of parents in Beijing believe that “childcare is necessary for all development,” and the proportion in Shanghai is as high as 95.3%. Liu Zhongyi's research results also show that at present, the parents of infants under the age of 3 in China have a strong demand for institutional care services. The demand for 0–3-year-old infant care services in urban areas is more prominent.

It is important to note that, packet loss ratio is defined as the ratio of the number of packets which are lost during the transmission to the total number of packets generated in the system, networks in this case. When the cycle length is 104 network packets, the false positive test results of malicious packet loss are shown in Figure 1. In the malicious packet loss false positive test, the horizontal axis of the experimental results in Figure 1 is the detection threshold. When the detection threshold of the system designed in this paper is about 0.25%, the occurrence probability of false positive approaches 0. The detection threshold of the original system needs to reach about 0.37%, and the occurrence probability approaches 0.

Under the same experimental environment, the false negative test results of malicious packet loss are shown in Figure 1.

In the false negative test, the random packet loss rate of abnormal nodes varies from 0.2% to 0.8%, and the cycle length is 105 network packets. As can be seen from Figure 2, while the packet loss rate of the two systems increases, the false negative rate decreases. When the packet loss rate of the original system is greater than 0.8%, the false negative probability is less than 2.0%. When the packet loss rate of the system in this paper is greater than 0.52%, the false negative probability is less than 2.0%.

The false positive test results of malicious packet modification of the two systems are shown in Figure 3.

In the test process, in the absence of malicious nodes, the probability of abnormal self-contracting caused by the network itself is 0.2%, and the cycle length is 104. When the sampling rate of the two systems increases, the probability of false positive decreases. In this system, when the sampling rate is 12.3%, the probability of false positive is 5%, and when the sampling rate in the traditional system is 50%, the probability of false positives decreased to 5%. It shows that the system designed in this paper can achieve a high safety level when the sampling rate is small.

The test results of malicious packet modification of the two systems are shown in Figure 4.

Finally, the false negative probability of malicious packet modification in the presence of abnormal nodes is tested. The threshold setting of the two systems is 0.4%. As can be seen from Figure 4, when the packet change rate is 0.4%, the probability of false negative is 1%, and gradually approaches 0 with the increase of packet change rate. When the packet change rate of the original system is 0.5%, the false negative rate gradually approaches 16%, on the other hand, it also verifies that the system in this paper has high accuracy in the intelligent location of network abnormal nodes.

## 6. Conclusion

In this paper, we have presented big-data-enabled methodology to ensure that proper and timely public childcare services are provided to every individual especially children both in the cities and the urban areas. These services are defined as the service required to be provided to a child when he/she interact with outside environment such as education. Moreover, these services must be ensured by the government especially through a dedication department. The statistical results show that people's demand for childcare services does exist. What also exists is the contradiction between people's demand for childcare and the insufficient construction of the number of childcare institutions and the single supply of the provider. This contradiction is the problem we urgently need to solve. If both husband and wife are the only children, compared with families with non-only children, the demand for childcare is lower, and the occurrence ratio of choosing childcare is 35.8%; the longer the family's working hours, the smaller the demand for childcare services. The above data show that the work and health status of grandparents in the family and the parenting concept of the two generations have an impact on the demand for childcare services. In addition, in families with more than two children, the greater the age difference between the second child and the youngest child, the less the demand for childcare services. For each additional year of age, the probability ratio of requiring childcare services to not requiring childcare services increases by 95%; the higher the respondents' psychological acceptance of childcare services, the greater the demand for childcare services; people who care about the facilities, environment, and food safety of nurseries have less demand for nurseries. [16–18].

## Figures and Tables

**Figure 1:** False positive test results of malicious packet loss of the two systems.

**Figure 2:** False negative test results of malicious packet loss of the two systems.

**Figure 3:** False positive test results of malicious packet modification of the two systems.

**Figure 4:** False negative test results of malicious packet modification of the two systems.

**Table 1:** The influence of parents having only one child on the choice of childcare services.

	1	2	3	4
Variable	if_*ty*	if_*ty*	if_*ty*	if_*ty*
The mother is the only child	−0.72 (0.49)	—	−0.42 (0.55)	—
Average family working hours per week	−0.02 (0.01)	1.12 (0.72)	1.23 (0.73)	1.24 (0.70)
Parents and grandparents take care of infants and young children	1.3 (0.75)	−0.02 (0.01)	−0.02 (0.73)	1.24 (0.73)
Grandparents take care of infants and young children	0.04 (0.02)	1.21 (0.13)	1.3 (0.7)	1.1 (0.21)
Observed value	175	175	175	175

**Table 2:** Impact of children's age difference on the choice of childcare services.

	1	2	3
Variable	if_*ty*	if_*ty*	if_*ty*
Maternal age	0.88 (0.42)	0.04 (0.20)	1.88 (0.45)
Age difference between the second child and the youngest child	0.02 (0.01)	1.42 (0.62)	1.23 (0.53)
Age of first child	1.5 (0.55)	0.02 (0.20)	0.23 (0.21)
Grandparents take care of infants and young children	0.04 (0.02)	1.21 (0.13)	1.3 (0.7)
Is the mother an only child	—	2.60 (1.18)	5.52 (2.16)
The father is the only child	—	−1.58 (0.03)	−2.1 (0.05)
Observer value	175	175	175
Observed value	60	60	60

**Table 3:** Influence of characteristics of nursery institutions on the choice of nursery services.

	1	2	3	4	5
	*E*1	*E*2	*E*3	*E*4	*E*5
Variable	if_*ty*	if_*ty*	if_*ty*	if_*ty*	if_*ty*
Distance between nursery institutions and Gao's family	-	-	1.30 (0.75)	-	0.25 (0.34)
Facilities, environment and food safety	-	-	-	-	−0.86 (0.35)
Quality of nursery clothes	-	-	-	-	−0.14 (0.24)
Nursery service qualification and reputation	-	-	-	-	−0.15 (0.36)
Psychologically acceptable charge level	0.76(0.38)	-	-	-	-
Personal or family care burden	-	0.77 (0.46)	-	-	-
Constant	0.97 (1.44)	2.34 (0.37)	1.53 (0.24)	1.53 (0.26)	0.57 (0.28)
Observed value	86	190	190	190	190

## Data Availability

The datasets used and analyzed during the current study are available from the corresponding author upon reasonable request.
